# Motor-Sparing Neural Ablation with Modified Techniques for Knee Pain: Case Series on Knee Osteoarthritis and Updated Review of the Underlying Anatomy and Available Techniques

**DOI:** 10.1155/2022/2685898

**Published:** 2022-05-31

**Authors:** Tony Kwun-tung Ng, King Hei Stanley Lam, Abdallah El-Sayed Allam

**Affiliations:** ^1^Pain Management Unit, Department of Anaesthesia and Operating Theatre Services, Tuen Mun Hospital, Hong Kong; ^2^Department of Anaesthesiology, LKS Faculty of Medicine, The University of Hong Kong, Hong Kong; ^3^Center for Regional Anesthesia and Pain Medicine, Wan Fang Hospital, Taipei Medical University, Taipei, Taiwan; ^4^Department of Anaesthesia and Intensive Care, Faculty of Medicine, The Chinese University of Hong Kong, Hong Kong; ^5^Board of Clinical Research, The Hong Kong Institute of Musculoskeletal Medicine, Hong Kong; ^6^Department of Family Medicine, The Chinese University of Hong Kong, Hong Kong; ^7^Department of Family Medicine, The University of Hong Kong, Hong Kong; ^8^Taiwan Association of Prolotherapy and Regenerative Medicine, Taichung, Taiwan; ^9^Department of Physical Medicine, Rheumatology and Rehabilitation, Tanta University Hospitals and Faculty of Medicine, Tanta University, Egypt; ^10^Morphological Madrid Research Center (MoMaRC), Madrid, Spain

## Abstract

Knee osteoarthritis (KOA) is ubiquitous. However, effective pain managements for patients with grades 3 or 4 KOA for whom conservative treatments are unsuccessful, but for whom surgery is not an option, remain lacking. This case series presented two motor-sparing interventional pain treatment modalities for five such patients. Three of the patients with a mean total WOMAC score of 41 underwent thermal radiofrequency (RF) ablation using a modified motor-sparing approach. One-week and four-week post-RF, the total score dropped to 27 (by 34%) and 19 (dropped 53.7%), respectively. Two other similar patients with a mean total WOMAC score 96 underwent chemical neurolysis using a motor-sparing approach with modified landmarks. The WOMAC score dropped to 58.5 (by 39.1%) and 49 (dropped by 49.0%), one-week and four-week postchemical neurolysis, respectively. A narrative review of the currently available approaches is also provided, with the conclusion that neural ablation using the modified landmarks approach may achieve better pain control and preserve the motor functions for patients with severe KOA for whom conservative treatment was unsuccessful and who are not candidates for surgery.

## 1. Introduction

Knee osteoarthrosis (KOA) is a very common joint disease, with a prevalence ranging from 4.2% to 15.5% and gradually increasing with age [1]. It was ranked 11th among the 291 disabling illnesses worldwide [2]. KOA is associated with diverse causes including age, obesity, metabolic bone diseases, and acute or chronic joint injuries [3]. Pain and disabilities are the major consequences of KOA, with 25% of patients suffering from severe arthralgia. KOA is believed to be a result of the failure of chondrocytes to maintain homeostasis between the synthesis and degradation of the extracellular matrix and from subchondral bone developing osteoarthrosis [4–8]. The treatment algorithm for KOA starts with noninvasive therapies such as medication, physical therapy, and rehabilitation. Patients in whom good pain control is not achieved may need minimally invasive procedures, ranging from intra- or periarticular injections to radiofrequency (RF) [8]. For KOA of grade 3 or higher, total joint replacement is still the standard of treatment option, unless the patient has contraindications for such surgery. Among the various interventional procedures, motor-sparing techniques, or genicular nerve blockade should theoretically provide an optimal balance between analgesia, early mobilization, and rehabilitation, as well as fewer complication rate. Here, we describe five cases of denervation by alcohol neurolysis or thermal radiofrequency in KOA and also put our observations in context by providing an updated review of the various motor-sparing techniques that are used to block or denervate the nerves supplying the knee.

## 2. Case Series

This case series describes and evaluates the outcomes of alcohol neurolysis and thermal RF ablation of the articular branches of the knee in KOA. Patients with KOA pain who underwent knee articular branch denervation via chemical neurolysis or RF ablation between April 2021 and Jan 2022 were included in this report. Institutional approval was sought from the New Territories West Cluster (NTWC) Research and Ethics Committee, Hospital Authority, Hong Kong (Reference no: NTWC/REC/21090).

### 2.1. Patient Population

Patients with severe KOA pain in public hospitals are usually referred to pain services for nonsurgical management when they are inoperable. Inoperability was defined as (1) unacceptably high risk associated with anesthesia as assessed by an anesthesiologist, (2) unacceptably high risk associated with surgery as assessed by a surgeon, or (3) patient refusal of surgery. Another reason for referral was the prolonged waiting time for total joint replacement. Between Apr 2021 and Jan 2022, all such patients presenting to the pain service of the public hospital were evaluated for knee joint denervation. The treatment modality was based on our institutional experience with satisfactory pain control with knee denervation. To be eligible for the denervation, patients had to fulfill the following criteria (as evaluated by the pain service): (1) radiographic confirmation of KOA of grade 3 or higher unresponsive to conservative treatments, (2) moderate-to-severe pain according to the patient or their caregiver, and (3) a positive diagnostic block (defined as an improvement of Western Ontario and McMaster Osteoarthritis (WOMAC) score ≥ 50%). The following exclusion criteria for knee denervation were also applied: (1) inability to assume a recumbent or semirecumbent position, (2) significant cardiac morbidity with hemodynamic instability, (3) respiratory failure requiring >50% O_2_ supplementation or assisted ventilation, (4) previous ipsilateral total knee arthroplasty or denervation, (5) concomitant lumbar spinal stenosis with lower limb radicular pain, (6) concomitant chronic hip and low back pain, (7) presence of significant psychiatric illness, or (8) significant coagulopathy (platelet count < 50, 000/mL or international normalized ratio > 1.5). Written informed consent for both the procedures and potential publications was obtained before all neuroablative procedures.

### 2.2. Procedure

At our institution, the motor-sparing neural ablation of the knee is accomplished using either alcohol neurolysis or thermal RF ablation. The anatomical basis for such neural ablation procedures was based on the recent cadaver studies by Tran et al. and by Fonkoue et al. [9–12]. The targets were the medial and lateral branches of nerve to vastus intermedius (NVI), the superomedial genicular nerve (SMGN), the infrapatellar branch of saphenous nerve (IPBSN), the inferomedial genicular nerve (IMGN), and the superolateral genicular nerve (SLGN). They were scanned by a linear probe (Samsung RS85 4-12 MHz linear probe). If patients presented with posterior knee pain, popliteal nerve plexus (PNP) would also be targeted by a high frequency curved probe (Samsung RS85 3-10 MHz curved probe). Diagnostic blocks were done under real-time ultrasound guidance whereas a combined ultrasound- and fluoroscopy-guided approach was adopted in each denervation procedure. 1–1.5 ml 1% ropivacaine was injected into each anterior target while 3 ml 1% ropivacaine was injected into the PNP for the diagnostic purpose. Patients generally were advised to have separate diagnostic and denervating procedures. For those who had significant traveling difficulties between their homes and our facility, we would have both diagnostic and denervating procedures done in the same session with the pain-provoking diagnostic test performed 10 minutes after the diagnostic blocks by passively flexing and extending the knee and with manual pressure. If a dynamic pain reduction of more than 50% is achieved, one can proceed to neurolysis with 1–1.5 ml absolute alcohol to each target. For alcohol neurolysis, 10 cm 22-gauge Quincke needles were used for all nerves except the IMGN, which was approached by a 5 cm or 10 cm Quincke needle of the same size depending on the thickness of the soft tissue layer. For thermal radiofrequency ablation, multitined expandable RF needles (5 or 10 cm Nimbus® RF needles) were used. The clinical criteria for determining denervation method are provided in Table 1.

For the medial or lateral branches of NVI, a high-frequency linear transducer was first placed longitudinally along the femoral shaft to look for the junction between the femoral shaft and its medial epicondyle. The accompanying superomedial or superolateral genicular artery should be identified as a guide to target the nerve. The transducer was then turned 90 degrees to provide a transverse view perpendicular to the femoral shaft. Using an in-plane approach, the RF needle was advanced percutaneously toward the area connecting the femoral shaft to the medial or lateral epicondyle (epiphysis/diaphysis junction) at the middle of the measured anteroposterior depth of the femoral shaft. The periosteum appeared as an echoic line running along the cortical bone. The RF needle was further advanced until the needle tip reached the fascial plane immediately above the periosteum. A supplementary coronal view allowed checking of the position of the needle tip close to the nerve and the vessel (Figure 1). The RF lesioning at this point could cover the medial or lateral branches of NVI.

The next target for RF was the adductor tubercle which was the true target for the SMGN. The transducer was placed in a coronal orientation over the medial femoral epicondyle and then slide proximally to the adductor tubercle. The target for RF was the bony cortex 1 cm anterior to the peak of the adductor tubercle, using an in-plane approach. This was often accompanied by the superomedial genicular artery. After denervating the SMGN, the needle could be further advanced beyond the adductor tubercle, and another denervation could be done 0.5–1 cm posterior to the peak of adductor tubercle. This was often accompanied by the saphenous branch of descending genicular artery (Figure 2).

At the superolateral side of the femur, two needle targets were needed to cover the relevant nerves. The first target was the junction between the femur shaft and the lateral epicondyle as the superomedial side. It covered the lateral branches of NVI (Figure 1). A supplementary coronal view could be used for needle tip checking. The RF needle was then redirected obliquely, about 45 degrees from the coronal plane, and advanced obliquely from anterior to posterior until the needle tip reached the junction between the posterior edge of the lateral femoral cortex and the superior edge of the lateral condyle. This was the target of the true SLGN (Figure 3).

To target the IMGN, the transducer was placed in a coronal plane over the medial femorotibial joint line and a long-axis linear slide distally to visualize the tibial enthesis of the medial collateral ligament. Once the nerve and its accompanying inferomedial genicular artery were identified, the transducer was then turned 90 degrees transverse to the axial orientation. Using an in-plane approach, the needle was advanced from anterior to posterior to fit at the midpoint of the tibial width, close to the periosteum. A supplementary coronal view allowed checking of the needle tip beneath the medial collateral ligament, close to the nerve and the vessel (Figure 4).

Posteriorly, using a curved probe, PNP could be ablated by putting an RF needle from lateral to medial in a supine position with the knee flexed at around 90 degrees. Three stacked radiofrequency lesions were created in the subcutaneous interspace between the popliteal artery and posterior knee capsule along the line joining the superior aspect of the two femoral condyles. If the chemical approach was adopted, the needle trajectory was modified such that the needle advancement was maintained underneath the lateral head of gastrocnemius and plantaris while the final needle position was the same (Figure 5).

### 2.3. Assessments

For quality assurance purposes, we assessed and documented each patient's pain scores and functional status before and after the intervention. The WOMAC is a common tool used to assess these impacts on patients with KOA. It has three domains (pain, stiffness, and function) and contains a total of 24 questions. Each question is rated between 0 and 4 depending on the severity.

The primary outcome measure was the total joint WOMAC pain score at 1-week and 1-month postintervention compared to that before the pain intervention. The secondary outcomes were the total WOMAC score, the total knee stiffness score in the WOMAC, the total functional score in the WOMAC, and the overall WOMAC score across the same time points. Adverse events were defined as unfavorable and/or unintended findings (including abnormal laboratory results) or symptoms associated with the study procedure, for instance, prolonged postprocedural pain and hematoma. All the postprocedural follow-ups were conducted by pain nurses in the pain clinic.

## 3. Results

The COVID-19 pandemic substantially disturbed the provision of elective pain service to chronic pain patients, leading to a small patient load during the current study period. Five patients fulfilled all requirements and were thus evaluated. Two patients underwent alcohol neurolysis while the other three underwent thermal radiofrequency ablation. The patient demographics are listed in Table 2.

The exact WOMAC scores of the patients are shown in Table 3.

Regarding the overall preintervention status, the mean total WOMAC score of all the five patients undergoing the modified motor-sparing neural ablative therapy was 63/96. One week after the neurolytic procedure, the total WOMAC score had reduced to 39.6/96 (drop by 37.1%) and further reduced to 31/96 (dropped by 50.8%) at 1-month postintervention. The overall mean pain score reduced from 15.6/20 before the procedure to 7.8/20 (dropped by 50%) and 5.8/20 (dropped by 62.8%) at 1-week and 1-month postintervention, respectively. The overall mean stiffness score had improved from 5/8 preoperatively to 2.4/8 (reduced by 52%) and 1.6/8 (reduced by 68%) measured at 1-week and 1-month postoperatively. The overall function score had improved from 42.4/68 preoperatively to 29.4/68 (improved by 30.6%) and 21.6/68 (improved by 49.1%) at 1-week and 1-month postintervention, respectively (Figure 6).

Clinical neurological examination of the lower limb was routinely performed after the denervation procedure. Neither motor nor sensory deficit was elicited in any recruited patient. On subsequent follow-ups, no wound infection was detected by the pain nurse in any recruited patient.

## 4. Context and Discussion

### 4.1. Innervation of the Knee Joint

Innervation of the knee joint follows Hilton's law, which states that the nerves supplying a joint also supply the muscles moving the joint and the skin over the joint [13]. The innervation of the capsule of the knee joint is divided into an anterior and a posterior group of nerves (Figure 7).

Sensory input for the anterior knee joint capsule [9] is carried by branches of (1) the femoral nerve (FN), through its muscular branches, the NVM, the NVL, the NVI, and the IPBSN; (2) the common fibular nerve (CFN) through its terminal articular/anterior branches, the SLGN, the inferolateral genicular nerve (ILGN), and the recurrent fibular nerve (RFN); and (3) the tibial nerve (TN) through the IMGN (see Figure 7). The superomedial quadrant is innervated by the SMGN, NVI, and NVM; the inferomedial quadrant, by IMGN and IPBSN; the superolateral quadrant, by the NVL, NVI, SLGN, and CFN; and the inferolateral quadrant, by ILGN and RFN; no articular branches from the obturator nerve have been found to supply the anterior knee joint capsule. There are anastomoses between these nerves and with the posterior group of the genicular nerves to innervate the entire knee joint capsule. Therefore, overlapping innervation from two or more genicular nerves is common.

Sensory input for the posterior knee joint capsule originates from the posterior division of the obturator nerve (PON), the sciatic nerve (SCN), the CFN, and the TN [10]. These branches form a plexus, the posterior genicular plexus or simply PNP, which is closely related to the popliteal vessels.

### 4.2. Denervation Techniques

Pericapsular denervation techniques for the major joints have opened new horizons for interventional pain physicians involved in the management of advanced osteoarthritis of the major joints. While regenerative injection therapy is proven to be useful in reducing pain and improving function in KOA [14–17], its value in advanced KOA remains questionable [18]. Denervation can serve as a continuum of the pain intervention spectrum.

### 4.3. Implications of the Current Case Series

We extrapolated our experience with alcohol neurolysis and thermal radiofrequency ablation in hip fractures or inoperable osteoarthritis of the hip to the management of advanced inoperable KOA [19–21]. The pain component of the WOMAC score was chosen as the primary outcome because it is usually the commonest assessment of the intervention efficacy in patients. The overall improvement that was approximately 70% in our patients implies that both modalities of denervation were effective in reducing pain. Morning stiffness improved markedly by 75% in our patients while the overall WOMAC score also improved by more than 50%, suggesting that the denervation procedure could improve patient's functional status, even though it did not modify the progress of joint degeneration.

Interestingly, the functional score was improved to a relatively smaller extent for both treatment modalities. This can be explained by the KOA severity. The patient who underwent alcohol neurolysis was often nonambulatory, and the resultant lower limb muscle wasting could be anticipated, thus a lesser impact on the functional score improvement. In patients who underwent thermal RF, the mean functional score was not high initially and, thus, was difficult to improve significantly. Moreover, a variety of other factors affect overall functional performance, such as altered biotensegrity secondary to joint deformity and chronic intracapsular inflammation.

In our patients, the overall benefit of alcohol neurolysis appeared to be noninferior to the traditional denervation by thermal radiofrequency ablation. No transient neuritis or an initial pain flare-up was detected in any of these patients 1-week postintervention.

## 5. Review of the Current Literature

Motor-sparing denervation/neuromodulation techniques for the knee joint are basically categorized into four main approaches. The earliest approach is to target the saphenous nerve or its infrapatellar branch. Pulsed radiofrequency is the usual neuromodulation technique applied, while thermal radiofrequency ablation or neurolysis are not used for this purpose. Cryoablation has also been described in this context. The most popular approach is to target the genicular nerves. However, recent cadaver studies revealed that articular innervation is far more complex [9, 10]. Despite this, thermal radiofrequency ablation, pulsed radiofrequency, chemical neurolysis, and cryoablation have been used to denervate these nerves [22–28]. Lastly, there is also some evidence for the use of intra-articular pulsed radiofrequency for knee pain [29, 30].

### 5.1. Saphenous/Infrapatellar Nerve

Neuralgia of the infrapatellar branch of the saphenous nerve is a pain generator in many patients with osteoarthritic knee pain [31, 32]. Identification of these nerves is done by using transcutaneous peripheral nerve stimulation, ultrasound, and fluoroscopy. However, most of the evidence comes from case series or case reports.

Cryoablation has also been used in this context [33, 34]. It is considered superior to thermal radiofrequency given the absence of postintervention neuritis and less procedural discomfort. A randomized controlled trial by Radnovich et al. showed that in patients with mild to moderate KOA, cryoneurolysis of the infrapatellar nerve resulted in significantly decreased knee pain and improved symptoms compared to sham treatment on days 30, 60, and 90 [33]. Among patients who demonstrated a continued benefit of treatment on day 120, those in the active treatment group maintained significantly improved WOMAC pain subscale scores on day 150 compared to the sham treatment group.

### 5.2. Intra-articular Pulsed Radiofrequency (IA pRF)

The rationale is to deliver an electrical field effect to the C fibers and, as a consequence, modulate the pain via the needle electrode positioned intra-articularly in the knee joint [30]. The pain-modulating effect of the electrical field in the joint is also thought to have the anti-inflammatory [35] protective effects and regenerative properties of IA cartilage. Yuan et al. compared the clinical effect of IA pRF on pain caused by refractory knee osteoarthritis with that of IA dexamethasone and found that pRF was significantly more successful than IA dexamethasone in relieving knee pain and reduction of synovial fluid concentrations of TNF-*α*, IL-1, and MMP-3 [36]. Gupta et al. performed a systematic review of published studies investigating conventional, pulsed, and cooled radiofrequency ablation in the setting of chronic knee pain, and they found that IA pRF was a safe and effective method, giving promising results up to 1 year of follow-up with minimal complications [28].

Aly et al. suggested that a specific technique and regimen of IA pRF consists of targeting the superolateral joint space by placing a linear probe on the upper outer border of the patella in the transverse axis [37]. A 5 cm short-beveled needle is advanced toward the center of the joint, via an in-plane approach, at an angle of 45 degrees to the skin. A diagnostic block is first performed by injecting 4 ml of diluted local anesthetic intra-articularly. Due to the potential chondrotoxicity of IA local anesthetics [38], they are not generally used during the procedure. However, local anesthetics can confirm the source of pain, thus offering a higher chance of success when combined with pRF. Unipolar pRF is applied at 42°C, a pulse width of 20 ms, and a voltage of 45-65 V for 15 minutes after inserting a G22 5 cm radiofrequency curved needle into the center of the joint.

Gulec et al. compared unipolar and bipolar IA pRF and found that bipolar IA pRF was more advantageous in reducing pain and improving function than the unipolar pRF 3 months after the intervention [39]. The technique involves inserting two 10 cm radiofrequency needles with 5 mm active tips at the medial and lateral sides of the patellar ligament until the tips are in the middle of the joint space in both the transverse and sagittal planes under fluoroscopic guidance. The distance between the two needle tips is adjusted to approximately 1 cm. Bipolar IA pRF is delivered at 42°C, a pulse width of 10 ms, and a voltage of 45 V for 10 minutes.

### 5.3. Genicular Nerves and RF in Other Articular Branches

There are 10 nerves that carry sensory input from the anterior knee capsule, and 4 nerves carry sensory input from the posterior knee capsule,

Early studies targeting the articular branches of the knee essentially tackled the genicular branches only, namely, the SMGN, IMGN, and SLGN. The ILGN is usually spared in view of its proximity to the fibular nerve around the fibula. These older studies used fluoroscopy as the only guidance, whereas the newer studies used either ultrasound guidance or combined ultrasound and fluoroscopy (CUF) guidance.

The initial technique of fluoroscopy-guided approach, as described by Choi et al., targets the SMGN, SLGN, and IMGN by looking for the periosteal junction between the shaft and the epicondyle of the corresponding long bone [40]. This is accompanied by sensory and motor stimulations. The threshold of sensory stimulation should be below 0.6 V. Due to anatomic variations, motor stimulation may be performed at 2.0 V and 2 Hz, while the absence of fasciculation is assessed in the lower extremity. Thermal RF ablation is then delivered in a standard manner.

Huang et al. reviewed eight publications including a total of 256 patients in their meta-analysis [41]. The authors concluded that ultrasonography was an effective safe, nonradiative, and easily applicable guidance method for RF for pain relief and functional improvement in osteoarthritis knee pain. The assessed studies also showed that targeting the genicular nerves achieved better pain relief than targeting intra-articularly or sciatic nerve. Other narrative and systemic reviews also concluded that radiofrequency treatments targeting the knee joint (the major or periarticular nerve supply or the intraarticular branches) had the potential to reduce pain from osteoarthritis or persistent postarthroplasty pain for a duration of 1 to 12 months [42, 43]; it is noteworthy, however, that most of the publications included in their review were nonrandomized trials. Mahmoud et al. compared the outcomes between fluoroscopy-guided and CUF-guided genicular ablation procedures and found that both guidance modalities led to marked improvements in pain scores and WOMAC scores, with the CUF group showing superior results to the group treated under fluoroscopy-guidance only [44].

In view of our recent understanding of the innervations of the anterior and posterior knee capsules, only targeting the SMGN, IMGN, and SLGN in denervation may be an oversimplified approach nowadays. In fact, the original landmarks for SMGN and SLGN only cover a few branches of these two nerves, and they actually mainly cover the medial and lateral branches of NVI [12]. The true target for SMGN is 1 cm anterior to the peak of the adductor tubercle [9, 11, 12]. Cadaver findings from both Fonkoue et al. and Tran et al. also found the IPBSN coursed just posterior to adductor tubercle [9, 11, 12]. Denervating IPBSN at this location may be safer than the superficial target as suggested by Fonkoue et al. because more surrounding soft tissues are present at this target [11]. This can reduce the risk of skin burn or irritation caused by denervation. It has also been reported that inadvertent internal skin burn is a rare but known complication after ablating the inferomedial genicular nerve [45]. The implication is that one should consider an RFA probe with shorter active tip in case of minimal subcutaneous tissues in this target.

Sensory stimulation indicative of intraarticular numbness or aching may be applied to improve the accuracy while motor stimulation can be considered to rule out any local muscle fasciculation and patellar twitching. However, this is not mandatory. The use of multitined expandable RF needles or cooled RF technique can maximize the lesion size. Stacked lesions can be created to improve nerve coverage, especially the PNP. Fluoroscopy in the true anteroposterior and lateral views can confirm the final needle position before denervation.

There was a theoretical concern that denervation at the adductor tubercle would lead to significant and prolonged flare-up because of the chemical/thermal injury to the tendon insertion of adductor magnus at the adductor tubercle. This could create iatrogenic tendinitis-like pain. However, such flare-ups were not observed in these five patients at 1-week postintervention. This might be explained by routine prescriptions of oxycodone and etoricoxib as the postintervention analgesics. When these analgesics are contraindicated, a short course of oral steroid is an alternative. Adjustment of the denervation target slightly proximal to the adductor tubercle so that the denervation process would be less likely to involve the tendon insertion can also be considered. However, further studies are needed to confirm this.

### 5.4. Chemical Neurolysis

Chemical neurolysis of the genicular nerves is also an option when radiofrequency facilities are unavailable, when the procedure is contraindicated, or when is a financial concern as reported by two patients who experienced satisfactory pain relief 6 weeks after the neurolytic procedure [23]. A mixture of 0.5 ml 1% lignocaine and 0.5 ml nonionic contrast is first injected to confirm the spread, followed by another 1 ml of absolute alcohol injection to yield a resultant alcohol concentration of approximately 50%. Phenol neurolysis has also been described and validated in a randomized controlled trial [25].

By extrapolating our experience in chemical hip neurolysis in inoperable hip fracture, 10 minutes of waiting time would be sufficient for evaluation of diagnostic knee articular branch blocks [19]. Injection of 3 ml of local anesthetic and 3 ml of alcohol is used to minimize the potential spread of neurolytic agent to the sciatic nerve and its main branches superficial to the popliteal artery. In contrast to thermal radiofrequency, a technical pearl to avoid the inadvertent spread of neurolytic agents to tibial and common peroneal nerves is to ensure that the needle trajectory is under the lateral head of gastrocnemius and plantaris so that the muscles can serve as natural barriers.

One of the biggest myths regarding knee denervation is the lack of optimal approaches. Given the 14 nerves involved in the knee joint innervation, it remains debatable whether partial denervation would be noninferior to complete denervation. It is also unclear how many and what nerves need must be denervated to provide adequate pain relief. We believe a modified, tailor-made approach would better fit individual needs.

This case series has some limitations, including its small sample size, nonrandomization of the denervation modalities, the absence of the control group, unblinded assessment, and the lack of postprocedure radiographic and electrophysiological assessments. The long-term effects of this modified motor-sparing neural ablation for knee pain are yet to be concluded. Further randomized controlled trials are warranted to validate the techniques more thoroughly.

## 6. Conclusion

Our case series suggested a modified approach of motor-sparing denervation for knee pain control in patients with KOA for whom other conservative treatments failed but who were not candidates for knee replacement. Our observations provided important insights to permit the suggestion of a modified motor-sparing denervation approach, by either a chemical or neuroablative way that hopefully optimizes the success rate and facilitates pain physicians to develop a tailor-made interventional algorithm in Kellgren-Lawrence classification grade 3 and 4 KOA management. Further randomized controlled trials are needed to validate the techniques described here more thoroughly.

## Figures and Tables

**Figure 1:** Nerve to vastus intermedius (NVI) denervation (either the medial or the lateral branches). (a) The transverse view shows the needle inserted in an in-plane approach to the midfemoral shaft. (b) The coronal view shows the Doppler signal that signifies superomedial or superolateral genicular artery at the junction of femoral shaft and femoral epicondyle. White arrow: needle; asterisk: the needle target. (c) A lateral view of fluoroscope of the knee with needle placement for NVI (either the medial or the lateral branches) denervation as shown at 1.

**Figure 2:** (a) Denervation of the infrapatellar branch of the saphenous nerve (IPBSN) posterior to adductor tubercle. (b) Denervation of superomedial genicular nerve (SMGN) anterior to adductor tubercle. Note the Doppler signals that signify the vessels accompanying the nerves. AT: adductor tubercle; white arrow: Nimbus® radiofrequency needle. (c) A lateral view of fluoroscope of the knee with needle placement for SMGN (more anterior) and IPBSN (more posterior) denervation as shown at 2.

**Figure 3:** Superolateral genicular nerve denervation. (a) An axial view to identify the posterior edge of the lateral femoral cortex manifested as an edge separating the lateral side and the posterior side of the cortex. (b) An oblique view at around 45 degrees from the coronal plane shows the femoral shaft. LFC: lateral femoral condyle; white arrow: the proposed needle trajectory toward the target point; asterisk: the final needle tip position when scanning from the oblique coronal plane to the axial plane.

**Figure 4:** Inferomedial genicular nerve (IMGN) denervation. (a) A coronal view shows that the IMGN and its accompanying inferomedial genicular artery are located underneath the medial collateral ligament with the needle tip shown. (b) A transverse view shows that the needle is inserted in-plane to the midshaft of the tibia. Solid white arrow: needle; hollow white arrow: medial collateral ligament. (c) A lateral view of fluoroscope of the knee with needle placement for IMGN denervation as shown at 3.

**Figure 5:** Popliteal nerve plexus neurolysis. (a) An ultrasound-guided lateral-to-medial needle trajectory underneath the biceps femoris, gastrocnemius, and plantaris. The final needle position targets at the intercondylar bony surface. BF: biceps femoris; G: lateral head of gastrocnemius; P: plantaris; LFC: lateral femoral condyle; MFC: medial femoral condyle; A: popliteal artery; bold white arrow: needle; thin arrow: needle trajectory. (b) The anteroposterior and the lateral views of the needle placement for the popliteal nerve plexus neurolysis.

**Figure 6:** The WOMAC score changes for patients underwent modified neural ablations. (a) The total WOMAC scores change. (b) The WOMAC pain scores change. (c) The WOMAC stiffness scores change. (d) The WOMAC function scores change.

**Figure 7:** The genicular nerves of the anterior and posterior knee. Courtesy of the NYSORA Nerve Block app: https://go.nysora.com/nerve-block-app/. CFN: common fibular nerve; TN: tibial nerve.

**Table 1:** Criteria for choosing the denervation method.

Thermal RF	Chemical neurolysis
Significant liver/renal impairment Dysrhythmia with suboptimal control Advanced cardiac failure (NYHA class 3 or above) Allergy to alcohol Patient preference	Presence of pacemaker, spinal cord stimulator, or intrathecal pump Advanced dementia Patient who desires a faster procedure or is intolerable to any lengthy procedure Unavailability of RF facility Patient preference

NYHA: New York Heart Association; RF: radiofrequency.

**Table 2:** Patient demographics.

Patient no.	1R	2R	3A	4A	5R
Age (year)	78	78	79	71	62
Sex	Male	Male	Female	Female	Male
Preintervention ambulatory status	Walk unaided with gait alterations	Walk unaided with gait alterations	Wheelchair outdoors; walk with cane indoors	Walk with sticks outdoors and indoors	Wheelchair outdoors; walk with cane indoors
KOA grading	Grade 3	Grade 3	Grade 4	Grade 4	Grade 4
Knee side	Left	Right	Right	Right	Left
Pain duration (years)	6	5	10	4	9
Denervation modality	Thermal RF ablation	Thermal RF ablation	Alcohol neurolysis	Alcohol neurolysis	Thermal RF ablation

KOA: knee osteoarthritis; RF: radiofrequency.

**Table 3:** Exact WOMAC scores of the five patients who underwent neural ablations.

	Pain			Stiffness			Function			Total		
	0 week	1 week	4 weeks	0 week	1 week	4 weeks	0 week	1 week	4 weeks	0 week	1 week	4 weeks
Pat 1R	14	3	3	3	1	0	17	10	10	34	14	13
Pat 2R	14	3	7	3	1	2	17	14	12	34	18	21
Pat 3A	20	4	6	8	2	2	68	23	32	96	29	40
Pat 4A	20	20	10	8	8	4	68	60	34	96	88	58
Pat 5R	10	9	3	3	0	0	42	40	20	55	49	23
Mean	15.6	7.8	5.8	5	2.4	1.6	42.4	29.4	21.6	63	39.6	31

## Data Availability

The data used to support the findings of this study are included within the manuscript.
